The article "Comparative molecular docking and molecular‐dynamic simulation of wild‐type‐ and mutant carboxylesterase with BTA‐hydrolase for enhanced binding to plastic" was retracted in 2022. Reasons: no approval from the institution; copyright claims.

# Comparative molecular docking and molecular‐dynamic simulation of wild‐type‐ and mutant carboxylesterase with BTA‐hydrolase for enhanced binding to plastic

**DOI:** 10.1002/elsc.202100083

**Published:** 2021-11-15

**Authors:** Fatana Lameh, Abdul Qadeer Baseer, Abubakar Garba Ashiru

**Affiliations:** ^1^ Department of Botany Faculty of Biology Kabul University Kabul Afghanistan; ^2^ Department of Biosciences Faculty of Science Universiti Teknologi Malaysia Johor Bahru Malaysia; ^3^ Department of Biology Faculty of Education Kandahar University Kandahar Afghanistan; ^4^ Department of Chemistry Zamfara State College of Education Maru Nigeria; ^5^ Green Chemistry Research Group Department of Chemistry, Faculty of Science Universiti Teknologi Malaysia Johor Bahru Malaysia

**Keywords:** in silico site‐directed mutagenesis, MD simulation, molecular docking, PETase, plastic

## Abstract

According to the literature review, microbial degradation of polyethylene terephthalate by PETases has been detected effective and eco‐friendly. However, the number of microorganisms capable of such feats is limited with some undesirable bioprospecting results. BTA‐hydrolase has been already reported capable of degrading polyethylene terephthalate. Therefore, mutation by in silico site‐directed mutagenesis means to introduce current isomer of PETase for polyethylene terephthalate degradative capability as a better approach to resolve this issue. This study aimed to use in silico site‐directed mutagenesis to convert a carboxylesterase from *Archaeoglobus fulgidus* to BTA‐hydrolase from *Thermobifida fusca* by replacing six amino acids in specific locations. This work was followed by molecular docking analysis with polyethylene terephthalate and polypropylene to compare their interactions. The best‐docked enzyme‐substrate complex was further subjected to molecular dynamics simulation to gauge the binding quality of the BTA‐hydrolase, wild‐type and mutant‐carboxylesterase with only polyethylene terephthalate as a substrate. Results of molecular docking revealed lowest binding energy for the wild‐type carboxylesterase‐polypropylene complex (‐7.5 kcal/mol). The root‐mean‐square deviation value was observed stable for BTA‐hydrolase. Meanwhile, root‐mean‐square fluctuation was assessed with higher fluctuation for the mutated residue Lys178. Consequently, the *R*g value for BTA‐hydrolase‐ligand complex (∼1.68 nm) was the lowest compared to the mutant and wild‐type carboxylesterase. The collective data conveyed that mutations imparted a minimal change in the ability of the mutant carboxylesterase to bind to polyethylene terephthalate.

**Abbreviations**
3D: 3‐dimension
AFEST: *Archaeoglobus fulgidus esterase*
Ala: alanine
Asn: asparagine
Asp: aspartic acid
Glu: glutamic acid
Gly: glycine
HI: hydropathy index
His: histidine
Leu: leucine
Lys: lysine
MD: molecular dynamic
Met: methionine
nm: nanometer
ns: nanosecond
PDB: protein data bank
PET: polyethylene terephthalate
Phe: phenylalanine
PP: polypropylene
Rg: radius of gyration
RMSD: root‐mean‐square deviation
RMSF: root‐mean‐ square fluctuation
Ser: serine
Thr: threonine

The article "Comparative molecular docking and molecular‐dynamic simulation of wild‐type‐ and mutant carboxylesterase with BTA‐hydrolase for enhanced binding to plastic" was retracted in 2022. Reasons: no approval from the institution; copyright claims.

## 1 INTRODUCTION

The high demand for plastics has seen its rising in daily life, such as in medical products, household goods, toys, personal care products, manufacture and so on. While plastic products make human life easier and bring comfort to daily life, they cause long‐lasting pollution to the environment as it takes hundreds to thousands of years for microplastics to decompose [1]. The issue is exacerbated by poor waste management and the lack of a proper recycling system of the products [1]. Exposure of plastic products to environmental chemicals, physical and biological conditions shreds the plastics into small pieces of nano plastics and microplastics with the diameter of (<100 nm) and (<5 mm), respectively [2]. Microplastic can be found in both terrestrial [3] and marine [4] environments.

Polyethylene terephthalate (PET) is among the most popular polyester in the market, among hundreds of other synthetic polymers. PET is polymerized from terephthalic acid (TPA) and ethylene glycol (EG), both of which are derivatives of crude oil. Persistence, stability, transparency, and low production cost are the main properties of PET that make it a highly utilized polyester worldwide [5]. Nonetheless, the same traits contribute to the slow degradation of PET [6]. Current methods to degrade PET are pricy, time‐consuming, produce other wastes into the environment. However, plastics' microbial biodegradation is more reliable and friendlier to rid plastics' from the environment [7]. Biodegradation sees microbes producing specialized enzymes to break down plastics into their small oligomers, dimers, or monomers. The monomers are then utilized as the microbes’ sole carbon and energy source [8]. Some microbial enzymes from family members of cutinase, lipase, and esterase can hydrolyze PET to some extent [5]. For instance, the *Thermobifida fusca* PET hydrolase is a cutinase that degrades the PET at a higher temperature [9].

In truth, the microbial‐assisted degradation of plastic is far from satisfactory, and the process is time‐consuming as extensive bioprospecting for effective microorganisms is required to do the job. A better way is to use existing microbial enzymes and tailor their enzymes to be partial in degrading plastics. For this purpose, the bioinformatics tools are the best approach for predicting biological mechanisms computationally while saving time and costs [10]. A good start to “create” a novel enzyme capable of degrading plastics is to mutate an enzyme from the member of the α/β‐hydrolase family, a family that PETase (PET hydrolase) also belongs. Our target enzyme is the carboxylesterase from *Archaeoglobus fulgidus* (AFEST), which exhibits high thermostability. [11]. Mutating the carboxylesterase to endow it with the degradative characteristics of a PETase is somewhat possible. The outcome considers the sequence and the 3‐dimensional (3D) structure of the enzyme being available in the literature [12]. Carboxylesterase is serine hydrolases whose structural and functional characteristics closely match the α/β hydrolase fold enzyme [11]. The catalytic mechanism of AFEST comprised a catalytic triad which consists of Ser160, His285, and Asp255. The AFEST structure has been successfully crystallized in complex with a sulphonyl derivative and deposited to the Protein Data Bank (accession code 1JJI) [12]. The most interesting feature of AFEST is its unusual spectrum of pH activity. The enzyme exhibited the optimal activity at 70 °C in pH 10‐11 and significant activity at pH 12. Therefore, this enzyme might be of particular °c interest for approaches involving directed evolution to generate valuable catalysts for industrial applications [11]. In silico site‐directed mutagenesis of AFEST can be performed to enhance and assess the enzyme's ability to degrade plastic compared to a well‐known PET hydrolase, the BTA‐hydrolase [13, 14].

The article "Comparative molecular docking and molecular‐dynamic simulation of wild‐type‐ and mutant carboxylesterase with BTA‐hydrolase for enhanced binding to plastic" was retracted in 2022. Reasons: no approval from the institution; copyright claims.

**PRACTICAL APPLICATION**

The high demand for plastics has seen its raising in daily life, the degrading process of plastics in the environment is a slow process; therefore, a method should be adopted to solve the issue. Mutation of the existing enzyme to enhance the degradability of plastic is the best approach that can be taken into consideration from the point of view of biotechnology. The current research can be applied by the companies and the design of the work gives the idea of mutation in other enzymes to speed up the degrading process and wipe out plastic waste.

## 2 MATERIALS AND METHODS

### 2.1 Structural preparation and multiple sequence alignment

The amino acid sequence of carboxylesterase from *Archaeoglobus fulgidus* (AFEST) was retrieved from Protein Data Bank (PDB) database (https://www.rcsb.org) PDB ID: 1JJI, Chain A [12, 15]. Meanwhile, the amino acid sequence of BTA‐hydrolase (plastic degrading enzyme) was also retrieved from the PDB database (PDB ID: 5zoa) Moreover, the enzyme commission number of both proteins was identified in Brenda e (http://www.brenda‐enzymes.org/).

The article "Comparative molecular docking and molecular‐dynamic simulation of wild‐type‐ and mutant carboxylesterase with BTA‐hydrolase for enhanced binding to plastic" was retracted in 2022. Reasons: no approval from the institution; copyright claims.

According to the literature, multiple sequence alignment (MSA) is applied to a set of algorithmic solutions of evolutionarily relevant sequences such as insertion, deletion mutation, and rearrangement under certain circumstances. DNA, RNA, or protein sequence may be added [16]. In this study, multiple sequence alignment included amino acid sequences of BTA‐hydrolase, wild‐type carboxylesterase (wild‐type AFEST), and mutant carboxylesterase (mutant‐AFEST) to highlight the mutant residues and compare the difference between them. The three above mentioned FASTA format of proteins was subjected to an online server of Multalin (http://multalin.toulouse.inra.fr/multalin/) in a single run. The residues to be mutated were selected randomly on the binding site of the sequence. Next, the already identified catalytic residues of AFEST were viewed using PyMOL, and the residues to be mutated were superimposed [17].

### 2.2 In silico site‐directed mutagenesis

The identified residues located on the conserved regions of the wild‐type AFEST seen in this study were believed to be involved in the binding site. The residues were substituted by in silico site‐directed mutagenesis [18], where six residues E34 (Glu), L82 (Leu), L121 (Leu), A169 (Ala), G178 (Gly), and D180 (Asp), on the chain A of the wild‐type AFEST was replaced with the corresponding N (Asn), T (Thr), F (Phe), M (Met), K (Lys), and A (Ala), respectively. The residues were proposed based on two factors of BTA‐hydrolase sequence and binding ability. The mutation was performed using PyMOL software by subjecting the protein's PDB file format [15]. Next, the molecular docking procedure was performed on wild‐type and mutant‐AFEST and BTA‐hydrolase with substrates to find and compare the proteins' highest binding affinity on the ligands.

### 2.3 Atomic composition and physicochemical properties

The primary structure (FASTA) of wild‐type AFEST, mutant‐AFEST, and also BTA‐hydrolase was subjected to ExPASy server through the Protparam tool (https://web.expasy.org/protparam/) to characterize their physicochemical properties [19]. The Protparam server was performed in a single run to obtain information, for instance, amino acid and atomic composition, formula, number of amino acids, molecular weight, theoretical Pi, the total number of negative and positive charges of residues, the total number of atoms of enzymes. Analysis and comparison of the evolutionary combinational changes and functional relationship among organisms can be made [20].

### 2.4 Structural validation

To validate the structure accuracy of mutant‐AFEST, the SAVES server's validation tools were used to assess the quality after mutation. The tools include PROCHECK [21, 22], ERRAT [23], and Verify‐3D [24] as validation indexes for models. The mentioned tools worked differently in the process of validating the reliability of the protein.

The article "Comparative molecular docking and molecular‐dynamic simulation of wild‐type‐ and mutant carboxylesterase with BTA‐hydrolase for enhanced binding to plastic" was retracted in 2022. Reasons: no approval from the institution; copyright claims.

### 2.5 Molecular docking

Molecular docking was carried out to establish the ligands' molecular interaction with the substrate binding residues of the BTA‐hydrolase, wild‐type, and mutant‐AFEST in the active site. This assessment is preliminary to compare the quality of interaction of enzymes with the tested substrates [10]. In this study, we focused on the docking of three proteins each one BTA‐hydrolase, wild‐type AFEST and mutant‐AFEST with the ligands, PET and PP. The retrieved PDB format of proteins is required to be used in docking. The 3‐dimensional structures of the ligands, polyethylene terephthalate (PET) (PubChem CID: 18721140) and polypropylene (PP) (PubChem CID: 32881) were retrieved from PubChem database (https://pubchem.ncbi.nlm.nih.gov) (3D modeling conformer) [25]. Then the SDF file format of the ligands was converted to PDB format using the BABEL program (version 2.3.1) [24]. Docking simulation, which included the blind docking method was employed using AutoDock version 4.2.6 and AutoTools 1.5.6 software to predict the active site on the three enzymes as mentioned above. In this step, water molecules were eliminated from the proteins, followed by polar hydrogen and non‐polar hydrogen. Next, the total Kollman and Gasteigher charges were assigned, respectively. The same procedure was imposed on the ligands to ensure that torsions for rotation were correctly adopted during docking. The grid box parameters were adjusted as ±1.000 Å spacing coordinating with sizes of 48, 50, and 50 of both wild‐type AFEST and mutant‐AFEST on the X, Y, and Z dimension, respectively. The grid box parameters were fixed with the size of 44 for three axes of X, Y, and Z for BTA‐hydrolase protein. Subsequently, the protein‐ligand complex was obtained in the PDBQT format [26].

Few independent docking runs were implemented on each ligand. Ultimately, the generated PDBQT file was analyzed by selecting AutoDock to identify the binding energy. The best result was gained for each substrate and protein based on the largest cluster of residues having the lowest binding energy [25]. The PDBQT format was then converted to a PDB file to be visualized by PyMOL and LigPlot to investigate protein and ligands interactions.

Consequently, the mutant‐AFEST was visualized by the software LigPlot for a clearer evaluation of the substrate biding residues' interaction with the tested ligands. Similarly, the wild‐type AFEST and BTA‐hydrolase interactions with the two ligands were represented using LigPlot software. The factors monitored are the hydrogen bond distance and the number of hydrogen bonds, and hydrophobic interactions in each enzyme‐ligand complex. LigPlot software is designed to describe the ligand‐protein schematic interaction as the 2D representation. Manual editing can be implemented on software, making it possible to provide different types of interactions such as hydrophobic and hydrophilic interaction [27]. The “pdbqt” file of each protein‐ligand complex was converted to “pdb” format using PyMOL and visualized in the LigPlot software.

The article "Comparative molecular docking and molecular‐dynamic simulation of wild‐type‐ and mutant carboxylesterase with BTA‐hydrolase for enhanced binding to plastic" was retracted in 2022. Reasons: no approval from the institution; copyright claims.

### 2.6 Model refinement

The generated 3D homology model of wild‐type AFEST, mutant‐AFEST, and BTA‐hydrolase were refined employing molecular dynamic (MD) simulation technique to confirm that the obtained native state was accurately at global energetic minimum [28], and the proteins are without major errors comparing to its native structure [29]. The parallel version of GROMACS 5.1.2 that employed the Gromos96 53a7 force‐field was used for MD simulation of proteins [30]. The hydrogens were added to the models so as the hydrogen bond network is broken in the water. This is because they tended to interfere with the protein structure [24, 31]. After refinement, the geometry of the refined 3D models was evaluated on the SAVEs (http://servicesn.mbi.ucla.edu/SAVES/) server by packages of ERRAT PROCHECK and Verify‐3D. To measure the dynamic behavior and structural modification, the root‐mean‐square deviation (RMSD) was also monitored for models refinement.

### 2.7 MD simulations for enzyme‐ligand complex

Stability of the docked complexes and interactions of BTA‐hydrolase, wild‐type and mutant‐ AFEST models with the selected substrate model of PET were investigated over a duration of 50 ns using the GROMACS 5.1.2 software for the proteins simulation which employed the force‐field 53a7 Gromos (http://www.gromacs.org/About_Gromacs). The topology and coordinate files of ligand and proteins were separately prepared to provide all the subsequent MD simulations' input files. The ATB server optimized the ligand (PET) for the system's contents [32]. The BTA‐hydrolase, wild‐type, and mutant‐AFEST proteins, and the ligand were merged using the energy minimized structures before continuing with the complex structure production run.

A 1.0 nm x 1.0 nm x 1.0 nm cubic simulation box simulated the proteins and the solutes while solvated in 180000 SPC/E water molecules for 50 ns under a constant temperature (300 K) and pressure (1.0 atm). The system's net charge was neutralized by adding counter ions, for which: 1 Na^+^ ion, 10 Na^+^ ions, and 7 Na^+^ ions were added to BTA‐hydrolase, wild‐type AFEST, and mutant‐AFEST to neutralize them. Under a mild condition, every system was applied energy minimization by using the steepest good algorithm up to a maximum of 10,000 steps and until the maximum force of (1000 kJ mol^−1^ nm^−1^) to eliminate steric clashes or inappropriate geometry [33]. Consequently, the MD simulations for the enzyme‐ligand complex were calculated via the root‐mean‐square deviation (RMSD), root‐mean‐square fluctuation (RMSF), and Radius of gyration (*R*g).

The article "Comparative molecular docking and molecular‐dynamic simulation of wild‐type‐ and mutant carboxylesterase with BTA‐hydrolase for enhanced binding to plastic" was retracted in 2022. Reasons: no approval from the institution; copyright claims.

## 3 RESULTS AND DISCUSSION

### 3.1 Structural analysis and multiple sequence alignment

The primary structure of a carboxylesterase (EC 3.1.1.1) from *Archaeoglobus fulgidus* (AFEST) assessed in this study has a total of 311 amino acids (PDB ID: 1JJI, Chain A). In contrast, the amino acid sequence of the BTA‐hydrolase (EC 3.1.1.101) from *Thermobifida fusca* (PDB ID: 5ZOA Chain A) contains 261 amino. Both sequences were obtained from the Protein Data Bank (PDB) database. Data revealed that AFEST is serine hydrolases.

In this part of the work, the amino acid sequences of BTA‐hydrolase and wild‐type AFEST were aligned by multiple sequence alignment using Multalin. This was done to identify important amino acids on the wild‐type AFEST based on the BTA‐hydrolase sequence, for site‐directed mutagenesis to introduce the ability in the mutant‐AFEST for plastic degradation. Overall, six residues were selected on the wild‐type AFEST binding sites to be mutated. Three of these residues were replaced based on the residues on the BTA‐hydrolase sequence, while three others were swapped by some hydrophobicity criteria and binding ability. Such as the residues Glu34, Gly178, and Asp180 on wild‐type AFEST were replaced with Asn34, Lys178, and Ala180 based on existence in BTA‐hydrolase sequence. On the other hand, three other residues Leu82, Leu121, and Ala169 were replaced with Thr82, Phe121 and Met169 respectively (Figure 1). The plastic's surface is hydrophobic, and its monomeric form, theoretically, would favorably form hydrophobic interactions [6, 34]. However, the extent of the hydrophobicity of residues Leu82 (Kyte‐Doolittle hydropathy index, HI = 3.8), Ala169 (HI = 1.8), and Leu121 on the wild‐type AFEST to affect the binding of PET to the mutant‐AFEST remains unclear. Hence, this study modulated the Leu82 (Kyte‐Doolittle hydropathy index = 3.8), Ala169 (HI = 1.8), and Leu121 on the wild‐type AFEST residues to less hydrophobic residues, Phe (HI = 2.8) and Met (HI = 1.9), and neutral residue Thr (HI = −0.7), respectively [35]. The reason behind of three aforementioned residues is that Methionine (Met) is believed to be important in the attempt to modulate mutant‐AFEST ability to bind PET, based on a report by Joo in year 2018 described that methionine assists in securing the PET in the enzyme's catalytic pocket through hydrophobic interactions [36]. In addition, Joo investigated the location of residues on different sites of cutinase (PET degrading enzyme) and it was confirmed that Phe is located at subsite II of the protein and plays role in the binding site. Moreover, Threonine (Thr) causes a conformational change of protein that causes the stability of the bound ligand to the active site [37].

The article "Comparative molecular docking and molecular‐dynamic simulation of wild‐type‐ and mutant carboxylesterase with BTA‐hydrolase for enhanced binding to plastic" was retracted in 2022. Reasons: no approval from the institution; copyright claims.

**FIGURE 1:** Sequence alignment of BTA‐hydrolase, wild‐type AFEST and Mutant‐AFEST. The black boxes show the mutation positions

In this study, wild‐type AFEST and mutant‐AFEST sequences belong to *Archaeoglobus fulgidus* species were aligned for comparison with the sequence of BTA‐hydrolase form *Thermobifida fusca* (Figure 1). AFEST contains the catalytic triad Ser160, His285, and Asp255 for sulfate reduction [12] that we did not perform any mutation on that region, as there isn't any prior knowledge of the AFEST's active site for plastic degradation. In the later part of the study, blind docking was conducted in the catalytic pocket of the mutant‐AFEST and compared to AFEST and BTA‐hydrolase to gauge differences in their binding affinity to PET.

### 3.2 In silico site‐directed mutagenesis

A protein's loops have been recognized as the most flexible regions than α‐helices and β‐strands. Therefore, replacing amino acids on a loop can significantly affect the structure and functional specificity [15, 38]. Considering that the catalytic triad of AFEST is formed by Ser160, His285, and Asp255 [12], these residues were not mutated. This is to avoid the canceling of the catalytic activity of the AFEST (Figure 2). In this study, an in silico site‐directed mutagenesis was done primarily on residues lining the catalytic pocket of the AFEST. We adopted this approach to convert AFEST into more BTA‐hydrolase‐like properties.

**FIGURE 2:** Comparison of wild‐type AFEST protein 3D structure with its mutant. (A) A 3D structure of AFEST protein superimposed with mutant‐AFEST and locations of mutated amino acids of E34N, L121F, D180A, and G178K on the front side view while L82T and A169M on the backside view. Red‐colored and blue‐colored sticks represent the wild‐type and mutant‐AFEST, while the grey‐colored depict superimposed wild‐type and mutant‐AFEST. Green labeled is showing the catalytic triad of protein, including Ser160, His285, and Asp255. (B) Individual 3D structure of AFEST before mutation and (C) after mutation

Data of multiple sequence alignment saw six residues Glu34, Leu82, Leu121, Ala169, Gly178, and Asp180 in AFEST mutated to match residues found on the same mentioned positions on BTA‐hydrolase, namely the Asn, Thr, Phe, Met, Lys, and Ala, respectively. Residues Glu34 and Ala169 are located on the front surface of alpha‐helix, Leu82, situated on a beta‐sheet strand facing slightly inside the protein. In contrast, the residues Leu121, Gly178, and Asp180 were sited on the outer loops (Figure 2A). The mutation with the targeted residues was quite agreeable because it was not expected to overly affect the mutant‐AFEST's structure and catalytic activity [15]. The overall surface outlook of mutant‐AFEST protein appeared to remain relatively unchanged (Figure 2C) compared to the wild‐type enzyme protein (Figure 2B).

The article "Comparative molecular docking and molecular‐dynamic simulation of wild‐type‐ and mutant carboxylesterase with BTA‐hydrolase for enhanced binding to plastic" was retracted in 2022. Reasons: no approval from the institution; copyright claims.

In our work, some moderate and relatively noticeable differences were detected in the molecular weight of residues related to the amino acids' substitutions as Glu34Asn, Leu82Thr, Leu121Phe revealed moderate differences, and Ala169Met, Gly178Lys, and Asp180Ala showed appreciable differences on the AFEST. Since the plastics tend for hydrophobic interactions [6], hydrophobic residues such as Phe, Met, and Ala residues were used in the mutations, while Thr was selected because of its neutral nature and mildly hydrophilic [35]. The in silico *s*ite‐directed mutagenesis performed using PyMOL affected only chain A of the AFEST protein. Validation of the mutant‐AFEST structure by PROCHECK, ERRAT, and Verify‐3D (Table 2) and results of physicochemical properties of three proteins are presented in Table 1. Moreover, mutations in enzymes are generally quite bearable if the substituting amino acids have a similar molecular weight [15, 39]. The next step of the study used blind docking to establish the best binding affinity for PET.

**TABLE 1:** Summary of physicochemical properties BTA‐hydrolase, wild‐type AFEST, and mutant‐AFEST identified by ExPASy's ProtParam

Details	Wild type‐AFEST	BTA‐hydrolase	Mutant‐AFEST
Amino acid residues	311	261	311
Molecular weight (Da)	35490.25	28174.62	35584.43
Theoretical pI	5.06	6.33	5.29
Negatively charged residues	46	24	44
Positively charged residues	34	22	35
Molecular formula	C_1602_H_2462_N_430_O_468_S_8_	C_1253_H_1945_N_347_O_384_S_5_	C_1607_H_2468_N_432_O_466_S_9_
Total number of atoms	4970	3934	4982
Aliphatic index (%)	92.51	80.80	90.00
Instability index (%)	42.71	36.02	42.70
GRAVY	−0.210	−0.229	−0.221

### 3.3 Atomic composition and physicochemical properties

The ExPASy server determined the physiochemical characteristics of proteins BTA‐hydrolase, wild‐type AFEST, and mutant‐AFEST via the Protparam tool (Table 1). Some main comparison of wild‐type AFEST and mutant‐AFEST is as following: generally, both has the same amino acid sequences 311 but difference in molecular weight, formula, total number of atoms. However, the new computed theoretical pI value for the mutant‐AFEST was 5.29, higher than the wild‐type AFEST at 5.06, likely due to the substitution of Glu34, Leu82, Leu121, Ala169, Gly178, and Asp180 residues to Asn, Thr, Phe, Met, Lys, and Ala of the wild‐type AFEST, respectively. It is indicated that a calculated theoretical pI value of below 7 implies acidic characteristics [19]. The computed wild‐type AFEST's instability index of 42.71 marginally reduced to 42.70 for the mutant‐AFEST. Both enzyme proteins remain intrinsically unstable (instability index >40) despite the mutation, probably due to certain dipeptides in the enzymes. This slightly reduced the aliphatic index of the mutant‐AFEST to 90.00 compared to 92.51 in the wild‐type AFEST. Note that an aliphatic index >40 implies a thermally stable protein; hence the mutations in this study only led to the slightly reduced thermal stability of the mutant‐AFEST [40]. The negative values of the grand average of hydropathicity (GRAVY) between the two proteins did, to a certain extent, produced a change with the wild‐type enzyme scoring a ‐0.210 compared to ‐0.221 in the mutant‐AFEST. The negative GRAVY values revealed their hydrophilicity, as the parameter indicates the protein's hydrophobicity and solubility. Conversely, a positive GRAVY value describes a hydrophobic protein [15, 41]. Notably, a lower GRAVY value of the mutant‐AFEST could be correlated to mutations of E34, L82, L121, A169, G178, and D180 to E34N, L82T, L121F, A169M, G178K and, D180A residues.

The article "Comparative molecular docking and molecular‐dynamic simulation of wild‐type‐ and mutant carboxylesterase with BTA‐hydrolase for enhanced binding to plastic" was retracted in 2022. Reasons: no approval from the institution; copyright claims.

Overall, the mutant‐AFEST collective data showing the higher pI value, reduced aliphatic index, and a more negative GRAVY value appear to be a step in the right direction for the study to convert the AFEST protein structure and characteristics to be more alike the well‐known PETase, the BTA‐hydrolase. However, the extent whether the site‐directed mutation‐related changes were adequate to improve the binding of mutant‐AFEST to PET remains to be seen. The in silico results are further discussed in the following subsections.

### 3.4 Structural validation analysis

The stereochemical quality of mutant‐AFEST was determined through PROCHECK. PROCHECK tool is used to investigate the stereochemical quality of protein structure based on the Ramachandran plot analysis and detailed residue‐by–residue listing [21, 33]. At least 90% of amino acids located within the most favored regions implying a good quality model [22]. The plot (φ‐ψ) represented mutant‐AFEST which shared the 89.1% number of residues in the most favored regions and was assessed protein of reasonable quality [22]. Residues in the additional allowed regions, generously allowed regions, and disallowed regions were detected 9.1%, 1.1%, and 0.7%, respectively.

The article "Comparative molecular docking and molecular‐dynamic simulation of wild‐type‐ and mutant carboxylesterase with BTA‐hydrolase for enhanced binding to plastic" was retracted in 2022. Reasons: no approval from the institution; copyright claims.

The phi (φ) and psi (ψ) values of the catalytic Serine (Ser160) were outside of generously allowable regions of mutant‐AFEST. This scenario is almost feasible, and literature dictates that catalytic Ser occurs rather often in disallowed areas in Ramachandran plots [42] (Figure 3). Furthermore, the overall quality factor score for mutant‐AFEST was scored 95.380 by ERRAT (Figure 4). ERRAT is valuable for verifying protein structures based on numbers of non‐bounded contacts within a cut‐off distance of 3.5 Å between different pairs of atom types (CC, CN, CO, NN, NO, OO). For a good model, an ERRAT score of >50% is considered reasonable [25, 33]. Consequently, the protein's compatibility with its own amino acid sequence was determined via establishing the Verify‐3D model. The Verify‐3D data showed that the model mutant‐AFEST scored 98.07% (Figure 5), since the standard range of score for the model is assumed to be >80% [25]. All in all, the enzyme 3D structures showed good quality and reliability for further structural analysis (Table 2).

**TABLE 2:** Results of structural validation of mutant‐AFEST proteins model with the SAVEs server

			Validation analysis%	
Validation	Parameter	Scheme	Mutant‐AFEST	Ranges scores (%)
PROCHECK	Most favored region (A, B, L)	Stereochemical quality	89.1	>90
	Additional favored (a, b, l, p)		9.1	
	Generously allowed regions [∼a,∼b,∼l,∼p]		1.1	
	Disallowed regions		0.7	
ERRAT		Overall quality factor	95.380	>50
Verify‐3D		Amino acid compatibility	98.07	>80

**FIGURE 3:** Ramachandran plots generated by PROCHECK showing a polypeptide backbone torsion angles psi (ψ) against phi (φ) of residues existed in the structures of mutant‐AFEST. The most favored regions [A, B, L] are colored in red. The additional allowed regions [a, b, l, p] are colored in yellow. The generously allowed areas [∼a, ∼b, ∼l, ∼p] are colored in pale yellow. All non‐glycine and proline residues are described as filled black squares, and glycine (non‐end) is shown as filled black triangles. The white color indicates residues in disallowed regions

**FIGURE 4:** The ERRAT validated an overall quality factor of the models for mutant‐AFEST. Yellow bars indicate the error regions between 95% and 99% and regions with a lower error are shown as white bars in protein folding

**FIGURE 5:** The outcome for Verify‐3D for mutant‐AFEST with the score of 98.07%

### 3.5 Molecular docking analysis

The PET and PP ligands' 3‐dimensional structures were retrieved in SDF format from the PubChem database (PubChem CID: 18721140) and (PubChem CID: 32881), respectively. PDB format files of wild‐type AFEST (PDB ID: 1JJI, Chain A) and BTA‐hydrolase (PDB ID: 5ZOA Chain A) were used for docking. PyMOL prepared the PDB format of proteins wild‐type and mutant‐AFEST, and only Chain A was employed in the docking study. The three other chains (B, C, D) of wild‐type AFEST and water molecule were deleted from the structure, while the BTA‐hydrolase only has Chain A. Literature has indicated that an enzyme's catalytic triad (active site residues) plays an important role in the biodegradation of substrate [43]. Previously, the catalytic triad of all types of PET‐hydrolase (PETase) was Ser160, His 237, and Asp206 [6, 36], and the BTA‐hydrolase also has the same residues as other reported PETases. The carboxylesterase, AFEST from *Archaeoglobus fulgidus* has a catalytic triad for sulfate‐reduction, comprised of Ser160, His285, and Asp255 [12]. In the current study, blind docking was performed as there isn't any prior knowledge on the active site pocket of the wild‐type and mutant‐AFEST [44]. In this research work, AutoDock Vina version 4.2.6 and AutoGrid tools 1.5.6 software were used for the docking analysis on PET and PP on BTA‐hydrolase, wild‐type AFEST, and mutant‐AFEST.

The article "Comparative molecular docking and molecular‐dynamic simulation of wild‐type‐ and mutant carboxylesterase with BTA‐hydrolase for enhanced binding to plastic" was retracted in 2022. Reasons: no approval from the institution; copyright claims.

Aside from observing for active site interaction between the enzyme‐substrates complexes, other parameters such as the highest binding affinity, hydrophobic interactions, hydrogen bonds, and hydrogen atom distance (Å) between an enzyme and ligand were also investigated. This is to provide a clearer insight and comparison into degradative mechanisms of the three tested enzymes [45]. The docking results of the BTA‐hydrolase with PET revealed two common residues Ser160 and His237, which previously formed hydrogen bonds with the substrate [6, 36, 46]. However, the docking outcome in this research revealed different positions for the interactions which occurred at Ser130 and His129. Another residue, the Ser66, showed the highest binding energy at (‐5.6 kcal/mol). This study seeks the lowest binding energy to identify the ligand's strong affinity with the enzyme, as previously indicated in the literature [47]. Results revealed that the lowest binding energy occurred for the wild‐type AFEST‐PP complex (‐7.5 kcal/mol), which resulted from one hydrogen bond formed with Ser160 at 2.91 Å. Table 3 summarizes the docking score for the protein‐ligand complexes with the corresponding hydrogen bond distance chosen as the highest binding energies for the different hydrogen bond interactions. Subsequently, the lowest binding energy was calculated for the mutant‐AFEST‐ PP (‐7.1 kcal/mol) with a shorter hydrogen bond distance of 2.84 and 2.87 Å with two amino acids Gln212 and Ser219, respectively. It is worth mentioning that the shorter the distance between two atoms, the hydrogen bond formed is stronger. As one of these two atoms acts as electron donor and the other one is electron acceptor [48]. The mutant‐AFEST‐PET complex showed lower binding energy (‐6.7 kcal/mol) than the wild‐type AFEST‐PET (‐6.3 kcal/mol), corroborated the mutations led to a stronger enzyme‐substrate complex. The mutant‐AFEST‐PET complex formed three hydrogen bonds with distances of 2.85, 2.99, and 2.71 Å to residues Tyr32, Gly89, and Ser160. Residues Tyr40 and Gly88 formed hydrogen bond distances of 2.92 Å, while the wild‐type AFEST‐PET complex formed triple hydrogen bonds to Ser160 at 2.79 Å and to residues Gly88 and Tyr40 at 2.88 Å. Interestingly, the docked BTA‐hydrolase ‐PP and BTA‐hydrolase ‐PET complexes formed remarkable weaker bonds that corresponded to ‐5.9 and ‐5.6 kcal/mol. BTA‐hydrolase ‐PP complex showed a slightly longer hydrogen bond distance of 2.96 Å to Ser130. The BTA‐hydrolase ‐PET complex's binding energy was comparatively the weakest bond with longest hydrogen bond distances of 3.21, 3.09, and 3.01 Å to Gly59 Ser66 and His129, respectively (Table 3). The shortest hydrogen bond distance was 2.71 Å, formed between mutant‐AFEST and PET.

The article "Comparative molecular docking and molecular‐dynamic simulation of wild‐type‐ and mutant carboxylesterase with BTA‐hydrolase for enhanced binding to plastic" was retracted in 2022. Reasons: no approval from the institution; copyright claims.

**TABLE 3:** Summary of docking analysis of BTA‐Hydrolase, wild‐type and mutant‐AFEST with two plastic substrates (PET) and (PP) from AutoDock Vina scores

		Hydrogen‐bond interaction		Hydrophobic‐bond interaction
Protein‐ligand complex	Score (kcal/mol)	Interacting residues	Distance (Å)	Interacting residues
BTA‐Hydrolase‐PET	−5.6	Gly59 Ser66 His129	3.21 3.09 3.01	Phe209, Tyr160, Asn212, Gly62
BTA‐Hydrolase‐PP	−5.9	Ser130	2.96	Met131, Trp155, His208, Gly59, His129, Phe209, Ser66, Gly62, Asn212
Wild‐type AFEST‐PET	−6.3	Tyr40 Gly88 Ser160	2.88 2.88 2.79	Ili92, Leu210, Phe218, Ile36, Ile209, Ile214, Lys22
Wild‐type AFEST‐PP	−7.5	Ser160	2.91	Val190, Phe193, Phe218, Leu210, Cys93, Tyr40, Asn289
Mutant‐AFEST‐ PET	−6.7	Tyr32 Tyr40 Gly88 Gly89 Ser160	2.85 2.92 2.92 2.99 2.71	Lys22, Ile92, Ile36, Leu210, Phe218, Ile209, Leu257
Mutant‐AFEST‐ PP	−7.1	Gln212 Ser219	2.84 2.87	Tyr40, Gly89, Cys93, Gly88, Ser160, Leu210, Phe218, Leu257, Val190, Met215, Phe193

Literature has shown that a longer hydrogen bond distance represents a lower affinity of the substrate to the enzyme, hence a more downward inclination to catalyze the compound [49]. This probably has to do with the plastic's hydrophobicity, which favors hydrophobic interactions between the enzyme and substrate [34, 50]. Figure 6 shows the LigPlot of the corresponding hydrophobic interactions of residues from the BTA‐hydrolase, wild‐type AFEST and mutant‐ AFEST bonded with the PET and PP substrates. Figure 7 portrays the LigPlot analysis for protein‐ligand interaction showing the formed hydrogen bonds with their equivalent distances.

The article "Comparative molecular docking and molecular‐dynamic simulation of wild‐type‐ and mutant carboxylesterase with BTA‐hydrolase for enhanced binding to plastic" was retracted in 2022. Reasons: no approval from the institution; copyright claims.

**FIGURE 6:** LigPlot analysis for protein‐ligand showing hydrophobic interaction with residues involved. (A) BTA‐Hydrolase‐PET, (B) BTA‐Hydrolase‐PP, (C) Wild‐type AFEST‐PET, (D) Wild‐type AFEST‐PP, (E) Mutant‐AFEST‐ PET and (F) Mutant‐AFEST‐ PP

**FIGURE 7:** LigPlot analysis showing the hydrogen bond interaction among proteins and ligands with its equivalent distance. (A) BTA‐hydrolase ‐PET, (B) BTA‐hydrolase ‐PP, (C) Wild‐type AFEST‐PET, (D) Wild‐type AFEST‐PP, (E) Mutant‐AFEST‐ PET and (F) Mutant‐AFEST‐ PP

### 3.6 Protein refinement and validation

Literature has shown that protein model refinement is necessary to ensure experimental consistency and prepare a protein model that is closer to its native structure [28]. Energy minimization is germane to eliminate any local strain and stabilize the structures into conformations closer to their native ones before substrate docking and molecular dynamic simulation [51]. For energy minimization, hydrogens are added to the protein models. This is because the hydrogen bond network is broken in water because it distorts the protein structure. The Root‐mean‐square deviation (RMSD) was calculated for mutant‐AFEST and the result showed that the model started to stabilize at 7 ns and 0.16 nm (1.6 Å) over the 50 ns production simulation. The model remained stable until 20 ns and fluctuated slightly upwards to 0.2 nm (Figure 8). According to Pandey [52] an acceptable range of RMSD value has a fluctuation between 0.2 and 0.3 nm, indicating protein is in a stable structure in terms of the protein's atomic position. Mutant‐AFEST was further evaluated by PROCHECK, which showed Ramachandran plots of 83.4% in the most favored regions, 14.4% in additionally allowed regions, 0.4% in generously allowed regions, and 1.8% in disallowed regions (Table 4). Therefore, the overall allowed regions were calculated 98.2%, which verified the mutant‐AFEST in a good quality model. The RMSD simulation result for mutant‐AFEST showed that the refined model was maintained stable during the 50 ns simulation with an average RMSD value of <0.3 nm. As a result, the refined models showed proteins of acceptable quality for further MD simulation investigations.

**FIGURE 8:** The plots of RMSD are depicted as a function of simulation during the time of 50 ns for refined mutant‐AFEST structures after energy minimization

**TABLE 4:** Results of structural validation of mutant‐AFEST protein model after refinement with the SAVEs server

			Validation analysis %	
Validation	Parameter	Scheme	Mutant‐AFEST	Ranges scores (%)
PROCHECK	Most favored region (A, B, L)	Stereochemical quality	83.4	>90
	Additional allowed regions (a, b, l, p)		14.4	
	Generously allowed regions [∼a,∼b,∼l,∼p]		0.4	
	Disallowed regions		1.8	
ERRAT		Overall quality factor	91.694	>50
Verify‐3D		Amino acid compatibility	96.14	>80

The article "Comparative molecular docking and molecular‐dynamic simulation of wild‐type‐ and mutant carboxylesterase with BTA‐hydrolase for enhanced binding to plastic" was retracted in 2022. Reasons: no approval from the institution; copyright claims.

### 3.7 MD simulations of the enzyme‐ligand complexes

This investigation is needed to analyze mutant protein's behavior versus the wild‐type or benchmark protein within a system. In this study, the geometrical quality of the Cα backbone–backbone conformation indicated the reliability of the enzyme was affirmed by the Root‐mean‐square deviation (RMSD) value to assess the conformational stability of a protein structure [53]. It is important to highlight that a relatively lower RMSD value (∼0.2‐0.3 nm) implies high stability of the complex structures and vice versa [52]. Since molecular docking results of wild‐type and mutant‐AFEST with PET only showed good satisfactory binding affinity of PET to the enzymes compared to the PP ligand; hence the MD simulation was performed only for PET.

The MD trajectory for the BTA‐hydrolase ‐PET complex showed fluctuations at 0.22 nm (2.2 Å) and then settled smoothly from 5 ns downward, with some minor fluctuations between 0.12 and 0.18 nm until the end of production simulation. On the other hand, the wild‐type AFEST‐PET complex reached equilibration at a slightly delayed time of 13 ns at an RMSD value of 0.18 nm. The trajectory remained relatively stable to the end of simulation at an RMSD mean of <0.25 nm. The mutant‐AFEST‐PET complex MD trajectory comparably fluctuated with RMSD values between 0.16 and 0.22 nm (1.6‐2.2 Å) that stabilized after 18 ns. The mutant‐AFEST‐PET complex displayed an overall RMSD below 0.25 nm implied a good enzyme‐ligand interaction. However, the BTA‐hydrolase‐ligand complex sustained better stability (under 0.2 nm) throughout the simulation. Interestingly, the wild‐type AFEST‐PET complex showed an average lower RMSD at 0.18 nm after 13 ns compared to the mutant‐AFEST‐PET complex (∼0.22 nm) at the same duration.

The result conveyed that the BTA‐hydrolase maintained a somewhat straight trajectory within low RMSD compared to mutant‐AFEST_PET, in which the latter demonstrated an upward fluctuation. The overall RMSD results between the three enzyme‐PET complexes indicate greater BTA‐hydrolase stability over the wild‐type and mutant‐AFEST (Figure 9). However, empirical studies are needed to clarify the in silico mutagenesis findings in this student. Hence they would merit an interesting investigation.

The article "Comparative molecular docking and molecular‐dynamic simulation of wild‐type‐ and mutant carboxylesterase with BTA‐hydrolase for enhanced binding to plastic" was retracted in 2022. Reasons: no approval from the institution; copyright claims.

**FIGURE 9:** Displaying the total RMSD plots as a function of simulation during the time of 50 ns complexed with PET. BTA‐hydrolase in green color, wild‐type AFEST in red color, and mutant‐AFEST in blue color

#### 3.7.1 Root‐mean‐square fluctuation (RMSF)

This research used RMSF analysis to discover knowledge on residue‐specific movement. During a simulation, RMSF measures each amino acid's flexibility and the extent of their fluctuation [24, 26]. A threshold value of RMSF of >0.05 nm (0.5 Å) identifies a remarkable change in residue‐specific flexibility [54]. The RMSF plots revealed the corresponding averaged RMSF values estimated for the BTA‐hydrolase ‐PET complex, wild type AFEST‐ PET complex, and the mutant‐AFEST‐PET complex was 0.05‐0.32, 0.05‐0.22, and 0.05‐0.43 nm. Hence, the wild‐type AFEST was more tightly bound to PET than BTA‐hydrolase about their average positions. The BTA‐hydrolase‐PET complex fluctuated the highest at Leu248 with an intensity of 0.32 nm, probably because it is on a loop. The BTA‐hydrolase catalytic triad, the Ser160, His237, and Asp206, positioned at the lowest fluctuation and bonded tightly to PET with RMSF values of 0.06, 0.1, and 0.07 nm. The wild‐type AFEST‐PET complex substantially fluctuated at Ile209 with an RMSF of 0.22 nm, again because of its location on the internal loop. Glu205 followed this at an RMSF value of 0.21 nm on an external loop. The mutant‐AFEST‐PET complex fluctuated the most for Lys178 with an RMSF value of 0.43 nm, where the residue is on loop region. The Gly204 residue on the BTA loop also exhibited an appreciable RMSF value of 0.3 nm (Figure 10).

**FIGURE 10:** The average RMSF is plotted as a function of the simulation time of 50 ns showing BTA‐hydrolase, wild‐type AFEST, and mutant‐AFEST against PET. BTA‐hydrolase is shown in green, the wild‐type AFEST in red, mutant‐AFEST in blue

Based on the study's RMSF data, the fluctuating Leu248 residue in the BTA‐hydrolase ‐PET complex, Ile209, and Glu205 in the wild‐type AFEST‐PET complex and Lys178 in the mutant‐AFEST‐PET complex were mainly located in the loop region. Fluctuations due to loops are assumed normal, considering these are the most mobile region in the protein structure [55]. The mutant residues, Glu34Asn, Ala169Met on the alpha‐helix region, Leu82Thr on the beta‐sheet region, and the Asp180Ala and Leu121Phe were located on loops occurred in the stable portion of the mutant‐AFEST‐PET. This enzyme‐ligand complex exhibited a low fluctuation in the range of 0.05‐0.1 nm. However, the only residue Gly178Lys fluctuated more at an RMSF value of above ∼0.3 nm (>3 Å), indicating poor interaction between the PET and the mutant‐AFEST. Since the mutation was performed in the binding sites and not in the catalytic triad, thus, residues Ser160, His285, and Asp255, mildly fluctuated with RMSF values within a reasonable range (∼0.05‐0.08 nm) [26, 56]. In all, the higher RMSF value observed in the mutant‐AFEST‐PET complex indicated a less stable enzyme‐substrate interaction compared to wild‐type AFEST‐PET complex and BTA‐hydrolase ‐PET complexes. As the loop region is usually the most fluctuating part of the protein, and it appears the substitution of Gly178 to Lys elevated the protein's fluctuation.

The article "Comparative molecular docking and molecular‐dynamic simulation of wild‐type‐ and mutant carboxylesterase with BTA‐hydrolase for enhanced binding to plastic" was retracted in 2022. Reasons: no approval from the institution; copyright claims.

#### 3.7.2 Radius of gyration (*R*g)

Compactional changes of the enzyme‐ligand complexes are measured by the radius of gyration (*R*g). Thus, this is considered a useful parameter to evaluate the protein structure's overall dimensions during MD simulation [57]. A folded structure with good stability is described by a fairly constant *R*g value. Conversely, an *R*g value that changes throughout simulation suggests an unraveled structure. A looser amino acid packing is reflected by a higher *R*g plot and vice versa [58]. In this investigation, the BTA‐hydrolase ‐PET complex fluctuated less at ∼1.68 nm. The enzyme‐ligand complex stabilized immediately after 5 ns, suggesting a well‐folded enzyme‐ligand complex structure [26]. *R*g plot for the wild‐type AFEST‐PET complex in contrast, fluctuated between 1.80 and 1.84 nm, which *R*g value is slightly higher than the BTA‐hydrolase ‐PET complex. The wild‐type AFEST‐PET complex achieved equilibrium from 28 ns onwards. Interestingly, the mutant‐AFEST‐PET complex also exhibited similar fluctuations as wild‐type AFEST‐PET complex with *R*g values ranging between 1.80 and 1.84 nm. The outcome seen here inferred a relatively stable interaction between the enzyme‐ligand complete despite the higher *R*g value. This indicated a less compact conformation of the wild‐type and mutant‐AFEST‐PET complex compared to the BTA‐hydrolase ‐PET complex [58, 59]. The study noted the *R*g plots for the wild‐type AFEST‐PET complex and mutant‐AFEST‐PET complex closely resembled each, thus a similar level of compactness between the two complexes. This agrees with their similar Rg values showing small fluctuations between 1.80 and 1.84 nm. From the *R*g overlay plot, the BTA‐hydrolase ‐PET's *R*g value was lower than both the wild‐type‐ and mutant‐AFEST‐PET complex (Figure 11). Hence, the BTA‐hydrolase appears to bind better with the PET than the two enzymes, suggesting mutations at residues Glu34Asn, Leu82Thr, Leu121Phe, Ala169Met, Gly178Lys, and Asp180Ala were not adequate to improve the change into a higher preference for PET. The findings also confirmed the earlier RMSD data, where the BTA‐hydrolase ‐PET complex was more stable than the mutant‐AFEST‐PET complex.

The article "Comparative molecular docking and molecular‐dynamic simulation of wild‐type‐ and mutant carboxylesterase with BTA‐hydrolase for enhanced binding to plastic" was retracted in 2022. Reasons: no approval from the institution; copyright claims.

**FIGURE 11:** The average gyration radius (*R*g) is plotted as a 50 ns simulation time function showing BTA‐hydrolase in green color, wild type AFEST in red color, and mutant‐AFEST in blue color complexed with PET

## 4 CONCLUDING REMARKS

This study explored the feasibility of converting a carboxylesterase from the *Archaeoglobus fulgidus* (AFEST) into a polyethylene terephthalate (PET) and polypropylene (PP)‐degrading BTA‐hydrolase equivalent from *Thermobifida fusca*. The study found six amino acids, Glu34, Leu82, Leu121, Ala169, Gly178, and Asp180, for possible mutation into the corresponding Asn, Thr, Phe, Met, Lys, and Ala. Molecular docking assessments of two different ligands, PET and PP, with enzymes, BTA‐hydrolase, wild‐type‐ and the mutant‐AFEST were done. The study revealed the wild‐type AFEST‐PP complex (−7.5 kcal/mol) gave the lowest binding energy, followed by mutant‐AFEST‐PP complex (−7.1 kcal/mol) and, lastly, the BTA‐hydrolase ‐PP complex with (−5.9 kcal/mol). The mutant‐AFEST showed lower binding energy (−6.7 kcal/mol) than BTA‐Hydrolase (−5.6 kcal/mol) when complexed with PET. Comparing the MD simulation data of the best docked mutant‐AFEST‐ligand structure against the BTA‐hydrolase ‐ligand complex revealed that the RMSD of the latter was stable between 0.12 and 0.18 nm after 5 ns. But the mutant‐AFEST‐PET complex equilibrated slightly later after 18 ns at ∼0.22 nm (2.2 Å). The corresponding RMSF value for mutant‐AFEST‐PET complex fluctuated the most for the mutated residue Lys178 at 0.43 nm, as the residue is sited on the loop region. In contrast, the loop‐sited Leu248 on the BTA‐hydrolase ‐PET complex exhibited the highest fluctuation with an RMSF value of 0.32 nm. The *R*g plots recorded a stable lower value of ∼1.68 nm for the BTA‐hydrolase ‐PET complex. Still, the mutant‐AFEST‐PET complex showed higher flexibility based on a higher *R*g value (∼1.80 and 1.84 nm) than BTA‐hydrolase ‐PET. In a nutshell, the six mutations on AFEST appeared to impart a minimal change in the ability of the mutant‐AFEST to bind to PET, based on molecular docking and MD simulation results. Probably, mutations of amino acids closer‐ and sited along the tunnel leading up to the catalytic site might yield better PET‐degrading ability into the mutant‐AFEST.

## CONFLICT OF INTEREST

The authors have declared no conflict of interest.

## ETHICS CLEARANCE

Human and animal data have not been used in the research.

## CONSENT FOR PUBLICATION

Authors agree to the publication.

## Data Availability

The data supporting the findings of the article is available in the [Protein Data Bank (PDB)] at [https://www.rcsb.org/structure/1JJI and https://www.rcsb.org/structure/5ZOA]; reference number [1JJI and 5ZOA]. Since the research is part of the thesis, data have not been shared.
